The article "Optimization of Management Structure and Resource Coordination Management Method of Construction Enterprises under Urban Environmental Pollution" was published in 2022. Journal: J Environ Public Health.

# Optimization of Management Structure and Resource Coordination Management Method of Construction Enterprises under Urban Environmental Pollution

**DOI:** 10.1155/2022/3823835

**Published:** 2022-08-10

**Authors:** Yan Xing

**Affiliations:** College of Urban Construction, Hebei Normal University of Science & Technology, Qinhuangdao 066004, China

## Abstract

The construction industry is an important pillar industry in China. It not only promotes the development of China's industry but also promotes the progress of society. It can be said that it has made great contributions to the development of China's economic construction. Issues such as sustainable development, green health, resource conservation, and environmental protection have become the most discussed topics, and it is imperative to implement green building management in the construction industry. Therefore, China has put forward the development concept of “green building,” which puts the management of green building on the basis of traditional building, and pays more attention to the goal of energy saving, environmental protection, people-oriented and green innovation. By studying the optimization of the operation structure of construction enterprises and the coordinated management of resources under urban environmental pollution, this study first observes the current situation of the construction industry this year and finds that the number of green building evaluation and identification projects in China is increasing year by year. Through in-depth analysis of management structure optimization and resource coordination methods, it is found that the first-level indicators have the largest weight in resource coordination management (E), followed by operation management (D), enterprise mechanism (A), talent quality (B), and management performance (C). The secondary indicator energy system planning and utilization (E2) has the largest weight value, followed by renewable energy utilization (E3), employee qualification rate (C1), waste management (D3), greening management (D2), energy conservation management (D1), main building energy conservation (E1), the impact of energy consumption on the environment (E4), management system (A1), corporate culture (A3), employee capability (B2), product quality pass rate (C3), intelligent system Management (D4), key brain drain rate (C2), talent atmosphere (A2), and employee quality (B1). Lastly, the first-level indicators have an impact on the operation structure of construction enterprises. The calculation results of the parameters are obtained to understand the impact of resource coordination management (E) on the operation of construction enterprises. In terms of enterprise mechanism (A), corporate culture (A3) and management system (A1) are relatively important reasons for affecting industrial resources; on talent quality (B) in terms of employee ability (B2), it has the greatest impact. Enterprises should pay attention to the introduction of talents and improve the comprehensive ability of employees. In terms of management performance (C), construction enterprises should train employees to improve their qualification rates. In terms of operation management, construction companies should pay attention to product quality (D), improve and optimize green buildings, and follow national policies and long-term development; in terms of resource coordination management (E), construction companies should continue to deepen the concept of green buildings, and at the same time strengthen the recyclability of green building materials and equipment, and the concept of recycling is still constant.

The article "Optimization of Management Structure and Resource Coordination Management Method of Construction Enterprises under Urban Environmental Pollution" was published in 2022. Journal: J Environ Public Health.

## 1. Introduction

Taking the recycling of construction waste in Central China as an example, this paper comprehensively studies the recycling of construction waste in developed regions (Europe and the United States). First, damage caused by urban construction waste polluting the environment was identified. Then, the environmental pollution caused by urban construction waste is analyzed, and the reasons for the obstacles to recycling and utilization of urban waste are summarized. Finally, the recycling measures for urban construction waste are put forward. The results show that the United States, Japan, and Germany have higher recycling rates of construction waste. The pollution of urban construction waste to the environment is reflected in the large-scale occupation of land resources, resulting in aggravation of household water, soil, and air pollution. The large amount of waste generated by large-scale urban construction and the low comprehensive disposal rate of construction waste are two aspects of urban construction waste pollution at present. The main reasons for the low recycling rate of urban construction waste are the lack of supporting laws, regulations, and industrial policies, the low market share of construction waste recycling products, poor coordination of key nodes in the industrial chain, and low operational efficiency. The research conclusions provide a good benchmark for improving the overall level of urban construction recycling development, promoting the sustainable development of construction waste recycling industrialization, and formulating construction waste recycling development policies and plans in other regions of China [1]. Based on the environmental statistics from 1992 to 2008, the changing trend, types, causes, and direct economic losses of domestic environmental pollution accidents were analyzed, and the risk areas of water and air pollution accidents were investigated using the SuperMap. The results show that the number of environmental accidents in 1994 was at most 3,001, and in 2007, the number was at least 462. The frequency of pollution accidents has decreased, especially after 2006. The most important accident types are all 54.3% and 34.2%. Pollution accidents are mainly production safety accidents and chemical transportation accidents, accounting for 30.8% and 26.9%, respectively. The heavily polluted areas are in the southeastern and central regions of China. Water and air pollution incidents occurred frequently in Guangxi, Hunan, Sichuan, and other places, and water pollution incidents in Zhejiang, Jiangsu, Guangdong, and other places occurred frequently. The direct economic losses caused by accidents mainly come from major accidents related to water pollution. Finally, recommendations are made for accident prevention and management [2]. The link coordination degree model is used to determine the coordination degree of environmental regulations, technological innovation, and green development. The city is divided into three systems: backward in the green economy, backward in environmental monitoring, and backward in technological innovation. Grey relational analysis is used to investigate factors influencing the development of the system. The three major eastern coastal cities, represented by Qingdao and Weihai, are well coordinated, while the development level of scientific and technological innovation, which is a key factor in the coordinated development of cities, is the lowest in Shandong Province. Grey correlation analysis shows that the development of green economy in backward cities has an impact on the level of economic development and foreign economic development; the impact of urban pollutant emissions is greater than the expenditure on pollution reduction when environmental regulation lags behind; the government's emphasis on personnel training is the technological innovation of backward cities. Based on these factors, recommendations for optimal urban development and coordinated regional development are formulated [3]. Urban environmental pollution and its governance are one of the issues that need to be explored in the development of modern cities. How to use relevant theories to analyze the current situation and causes of urban pollution, study pollution prevention, and control countermeasures, and achieve the coordination of urban development is of great significance and feasibility for the development of China's urban environment [4]. Shanghai's current environmental management framework, built on a post-transition socialist economy and spectacular urban renewal, has succeeded in reducing severe industrial pollution and improving urban facilities in unprecedented ways. However, it generally does not consider issues such as social and environmental justice. Based on Holden's sustainable urban development model, four priorities and five principles for Shanghai's future environmental management under the fair and shared city model are proposed, and their policy implications and implementation issues are briefly discussed. Horton's approach is relevant to the Shanghai case because he believes that the principle of multidimensional justice is central to the concept of sustainable development [5]. Systematic research is being carried out on the environmental pollution caused by the engineering structures ubiquitous in Chinese cities. Combined with the construction practice and the concept of environmental pollution control, a comprehensive method to prevent and control this problem and a calculation method of the Environmental Pollution Index (EPI) are proposed. Combined with the EM ISO14000 series of standards and relevant Chinese regulations, a civil engineering environmental pollution management system has been established [6]. The environmental pollution risk management assessment of Musayyib Power Station defines the coordination degree and response methods of the competent authorities in the field of environmental pollution monitoring. For research purposes, 150 individuals with no probability were selected as a sample, and a two-part questionnaire was used to collect data; and including demographic data and environmental pollution risk management, a total of 26 papers were collected. Local governments collect data from power plant workers and analyze it using applied statistical, descriptive, and inferential methods. The results showed that most of the participants were in the age group (25–35 years old) and most of them were male. In the field of education, most of them are formally graduated and work in administrative jobs without training in this area. Likewise, the results describing the results (70.7%) disagreed with the fact that there was a risk of environmental pollution, and there was a significant relationship between risk management and the level of education and training of the participants [7]. The time series data of Hefei City were selected from 2007 to 2014, and the objective weighting method was used to calculate the weight of the six indicators of urban pollution, and to examine the impact of urbanization on urban pollution. According to the results of the data stability test, a nonlinear model of the relationship between population urbanization and urban environmental pollution is established. The quadratic regression model fits well, and the intensity ratio also increases, indicating that there is a strong positive correlation between the two variables. Further regression analysis shows that the impact of population urbanization on urban environmental pollution is more obvious. Compared to the EQR curve, it shows the reason for the lack of an “inflection point” in the urbanization process. Finally, some suggestions are put forward on how to realize the coordination of population urbanization and urban environmental protection in Hefei in the future [8]. In order to strengthen the guarantee function of safety management organization for production safety and improve the safety level of construction enterprises, by analyzing the disadvantages of traditional construction enterprise safety management organization structure in technical practice, and carrying out structure-based optimization methods, the modern enterprise organization theory is put forward. The degree of orderliness is used as an indicator for evaluating the organizational structure of safety management. Time yield entropy and quality entropy are considered two dimensions of evaluation. Based on the entropy theory, an evaluation model of the order degree of the safety management organization structure is established. Take a state-owned enterprise as an example. By comparing the organizational structure of safety management with the degree of order before optimization, the method of the optimization scheme is verified. The results show that the orderly and optimized safety management organizational structure has been significantly improved, and the optimized safety management organizational structure has obvious advantages over the original organizational structure [9]. Environmental pollution and resource scarcity are two major challenges facing the world today, and the development and utilization of precious metal resources are one of the effective strategies to deal with these problems. Known for their high performance and scarcity, precious metals are essential in today's life. As a non-renewable resource, the demand and consumption of precious metals are increasing year by year. Therefore, it is imperative to develop eco-efficient precious metal recovery technologies to alleviate the environmental and raw material crisis. This perspective summarizes some common precious metal recovery strategies, focusing on innovations from traditional technologies. The above methods are evaluated and tested in terms of secondary pollution and recovery efficiency [10]. Given the conflicting nature of the resource and environmental issues, a new approach is needed. In this context, finding common ground and cooperation is expected to become a paradigm for conflict resolution. Economists can help design institutions that promote these paradigms. In order to control pollution, the common ground paradigm states that polluters and victims jointly decide emissions, pollution control, and financing. For pollution management, a new policy tool is proposed, including taxes, subsidies, and cost-sharing. Using this tool, the coordination process involves the Consensus between polluters and victims. The decision to discharge and reduce pollutants [11]. Use the VAR model to analyze the relationship between data stability, economic growth, and environmental pollution: emissions to the atmosphere, industrial sewage, and industrial solid waste. Solid waste the impact of industrial waste and the discharge of industrial waste in flue gas has been delayed, but it is still related. The increase of SO_2 affects economic growth to a certain extent, but it does not rule out that the government will play a role in the production process, industrial solid waste, industrial wastewater discharge, etc. The degree of supervision and innovation in aspects of the city. The impact of emissions on GDP is not significant [12]. Based on the location of urban road construction dust pollution sources and the optimization of urban road construction dust pollution emission reduction efficiency, an urban road construction dust source distance detection model was developed. Urban road construction uses remote sensing image technology to detect dust pollution of urban road structures, perform multi-level and multi-directional segmentation of remote sensing images, and use spatial block area matching to demarcate the visual features of suspicious buildings. The simulation results of the location of dust pollution sources in expressway construction show that this method is more intelligent and accurate in the positioning of urban dust pollution sources, and solves the problem of large errors in traditional manual positioning [13]. The environmental ratio quantifies the evolution of each industry and its impact on the environment. The evolution of the industrial structure has had a significant impact on these natural ecological environments, and the optimization of the industrial structure has not changed the dependence on natural resources and the ecological environment, so the research field should optimize the industrial structure, and improve the industrial structure. The utility effect of natural resources reduces various types of pollution and limits the impact of industrial structure buildings on the ecological environment [14]. Real-time dynamic optimization method of construction project progress based on lean construction the method is based on the process of construction companies Reengineering and Lean Supply. The newly proposed lean forecasting method uses multiple linear regression, back-propagation artificial neural network, and learning curve; considering the limited resources and constant project duration, the real-time dynamic programming optimization method adopts the resource-based concept. An intelligent schedule is a developed management system to optimize the progress of construction projects in a timely and efficient manner. The initial schedule can be programmed, and the dynamic real-time schedule can be optimized and displayed in Gantt charts, network charts, and spatiotemporal line charts [15].

The article "Optimization of Management Structure and Resource Coordination Management Method of Construction Enterprises under Urban Environmental Pollution" was published in 2022. Journal: J Environ Public Health.

## 2. Management Structure Optimization and Resource Coordination Management of Construction Enterprises under Urban Environmental Pollution

### 2.1. Current Status of Environmental Protection Management

Through the research and analysis of relevant civil engineering cases, it can be concluded that many construction units do not pay attention to environmental management when carrying out construction operations. Therefore, the adverse effects of construction are becoming more and more serious, and problems such as noise pollution cannot be truly solved. Affected by various aspects, the living conditions of urban residents have deteriorated sharply, and the construction units cannot achieve the expected economic benefits. During the construction of engineering structures, there are some water, air, and noise-related nuisances. These pollution problems pose a serious threat to the urban environment and negatively impact human health. Although construction units have begun to pay attention to environmental management in civil construction, their environmental management is not perfect due to various practical factors. Among them, lack of advanced environmental management techniques of the construction unit is an important reason affecting its project progress. In the process of governance and prevention of building pollution problems, the full function of pollution control equipment is more important. Today, most construction units mainly use old-fashioned cleaning equipment when dealing with pollution problems. The efficiency of these devices cannot meet the actual needs of the current pollutant purification work, so the purification work efficiency is low, as shown in Figure 1.

Many construction units do not pay attention to environmental protection management when carrying out construction work. As a result, the adverse effects of its construction have become increasingly serious, and problems such as noise pollution cannot be truly solved. Under the adverse effects of various aspects, the living conditions of urban residents have declined significantly, and construction units have therefore not been able to obtain the desired economic benefits. In the process of treatment and prevention of pollution problems in civil construction, whether the functionality of the equipment used for pollution treatment is complete occupies a larger position. At present, most construction units mainly use old-fashioned treatment equipment when dealing with pollution problems.

The article "Optimization of Management Structure and Resource Coordination Management Method of Construction Enterprises under Urban Environmental Pollution" was published in 2022. Journal: J Environ Public Health.

### 2.2. Characteristics of Urban Environmental Pollution Caused by Construction Products

Urban construction waste is often mixed with urban domestic waste. The pollution of urban domestic waste is dominant. Ordinary people can feel it with the help of sight and smell. Construction waste usually does not directly cause people's sensory response, which weakens people's perception of it. The city's cognition and awareness of the hazard of construction waste often lead people to ignore the specific impact of construction waste. In addition, the secondary characteristics of urban construction waste transportation cause the environmental impact of urban construction waste to be temporary. Small new buildings have a limited environmental impact as the number and size of buildings increase, and serious ecological and environmental problems often become more apparent. When distinguishing between construction and finishing materials, some products may contain large amounts of hazardous substances such as paints and coatings, and the release of these toxic substances has a lasting impact on the environment. Construction sites are easily polluted during the transportation of building materials and have the characteristics of large impact and large area. Building products can cause different levels of environmental pollution, from the production of building materials to the use and scrapping of building products. Sudden environmental pollution occurs when hazardous substances leak into building materials; when buildings collapse due to earthquakes, strong winds, and heavy rainfall, or when building products are dismantled at the end of their useful lives. Dusty materials (cement, lime, etc.), broken packaging bags, flying dust, paint and other materials, and fire will concentrate the harmful substances in the evaporation of paint, which will severely pollute the environment. It is shown in Figure 2.

1. Extensive
2. Ambiguity
3. Hysteresis
4. Sudden
5. Durability

The article "Optimization of Management Structure and Resource Coordination Management Method of Construction Enterprises under Urban Environmental Pollution" was published in 2022. Journal: J Environ Public Health.

### 2.3. Optimization of Construction Enterprise Management Structure under Urban Environmental Pollution

The competent department should first adjust the work attitude and realize the positive impact of environmental management during the construction period on the urban environment. After the relevant departments inform the relevant environmental protection staff, they should continue to increase publicity efforts so that all staff on the construction site can recognize the importance of effective environmental management to the construction unit and society. In the process of proper environmental protection publicity and education, environmental protection workers can put up advertising posters on the construction site. The advertising content should focus on the harm of construction pollution to urban residents, the environment and civil engineering, and let more construction workers explain the importance of its implementation. Relevant environmental management personnel should actively learn more advanced and effective environmental management technologies, and use these technologies to improve and optimize their own environmental management in civil construction. When carrying out appropriate management work, effective management of building materials for civil buildings can reduce the pollution of the building environment to the urban environment to a certain extent. Relevant construction units should strictly control the quality and safety of building materials to ensure that the building materials they use meet national requirements. Construction units actively use building materials that are compliant and less polluting, which to a certain extent helps to effectively control pollution sources in the structure. When carrying out work in the field of environmental protection management, relevant construction units must strictly abide by the legal requirements and standards related to environmental protection management. At the same time, the environmental protection management workflow should be explained in detail in the bidding documents when the project is tendered and tendered, and the relevant departments should be asked to supervise. This kind of behavior can enhance the self-management awareness of civil engineering units and make them restrained in further environmental management work. Self-control is also important in the supervision of environmental management. When managing construction materials and civil engineering pollutants, relevant personnel should ensure that their materials and equipment comply with environmental management requirements. At the same time, avoid the use of outdated equipment or highly polluting building materials, so as not to exacerbate the urban pollution problem, as shown in Figure 3.

1. Strengthen environmental protection publicity for the company's personnel, so that the environmental protection awareness of all employees can be improved;
2. Optimizing the implementation strategy of environmental protection management;
3. Learn advanced environmental protection management technology and continuously introduce new equipment;
4. Effectively supervise the environmental protection management process.

The article "Optimization of Management Structure and Resource Coordination Management Method of Construction Enterprises under Urban Environmental Pollution" was published in 2022. Journal: J Environ Public Health.

### 2.4. Coordinated Management of Resources under Urban Environmental Pollution

Analyze and solve the contradiction between resource development and urban construction from the perspective of sustainable development. Resource development must adapt to the carrying capacity of the environment in order to form a vicious circle and achieve sustainable development. This requires the formation of a vicious circle of urban construction, environmental protection, and resource conservation in the process of developing urban resources to create conditions for long-term development. The circular economy is an economic growth model based on resource efficiency and reuse, based on the principle of “resource reduction, reuse and utilization,” with low consumption, low emission, and high efficiency as the core features are the resource-based city. In order to build a harmonious society and achieve sustainable and healthy development, Huolin Gol City must take the concept of circular economy as the guideline for the next few years, formulate special plans for circular economy development, promote circular economy plans, and formulate and implement circular economy promotion plans for local economy. They should also develop laws and regulations and preferential policies for finance, taxation, etc., guide and support the development of circular economy, and strengthen the comprehensive utilization of resources and the utilization of circular economy in terms of resource extraction, production and consumption, and waste and social consumption. From the past one-way linear “resources, products, waste” mode to the “resources, products, renewable resources” multidirectional circular economy mode, sustainable development realizes the preservation of resources, products, and renewable resources, and realizes the “mutual promotion and win-win” of economy and environment.

The classification, recycling, and reuse of construction waste is an optimized plan for material-saving measures. The green construction of construction projects should focus on environmental protection, water saving and water resource utilization, conservation and material resource utilization, energy saving and energy utilization, land conservation and land resource protection, etc. Five aspects are evaluated in such an approach. In order to avoid the situation that the supervision is not in place in the project, corresponding measures are formulated to strengthen the supervision of each link.

The article "Optimization of Management Structure and Resource Coordination Management Method of Construction Enterprises under Urban Environmental Pollution" was published in 2022. Journal: J Environ Public Health.

## 3. Experimental Models

### 3.1. Analysis Method of Grey Relational Degree

Due to the different units of measurement for each factor and the different sizes and orders of magnitude of the original data, the different sizes and orders of magnitude are not easy to compare, or it is difficult to draw correct conclusions when comparing. Therefore, the raw data is usually subjected to dimensionless processing before the correlation is calculated.

Since each factor has different units of measurement, the original data have differences in dimension and order of magnitude. Different dimensions and orders of magnitude are not easy to compare, or it is difficult to draw correct conclusions when comparing. Therefore, before calculating the correlation degree, the original data is usually subjected to dimensionless processing.

The initialization is to remove all subsequent data from the first data using the same sequence to obtain multiple sequences of each data relative to the first data. In general, the baseline method is suitable for underestimating relatively stable socioeconomic phenomena, since most of such series are suitable for stable upward trends, and the treatment of the baseline values can make the upward trend more pronounced. For example, the launched series includes a dynamic development rate index commonly found in socioeconomic statistics. The general formula is:

(1) $$\begin{array}{c} y=\frac{x_{i}}{x_{0}}. \end{array}$$

The determination is to first get the mean of each original series, and then divide all the series data by the series mean to obtain multiple series of dynamic means for each data pair. Generally speaking, the averaging method is more suitable for data processing without obvious upward and downward trends. The general expression is:

(2) $$\begin{array}{c} y=\frac{x_{i}}{\bar{x}}. \end{array}$$

To cite a reference series refers to a data system used as a standard or basis. It can be dynamic or static. Let the reference number column after data processing be:

(3) $$\begin{array}{c} \left\{x_{0}\left(t\right)\right\}=\left\{x_{01},x_{02},\cdots ,x_{0n}\right\}. \end{array}$$

The *P* number sequence structures compared with the reference sequence structure are:

(4) $$\begin{array}{c} {\left\{x_{1}\left(t\right),x_{2}\left(t\right),\cdots ,x_{n}\left(t\right)=\left[\begin{array}{cccc} x_{11} & x_{12} & \cdots & x_{1n}\\ x_{21} & x_{22} & \cdots & x_{2n}\\ \vdots & \vdots & \cdots & \vdots \\ x_{p1} & x_{p1} & \cdots & x_{pn} \end{array}\right]\right\}}_{p\times n}. \end{array}$$

In formula (4), *x*-data value, *i*-the ith object, *t*-period *t*, *j*-jth indicator; when *i* = 0, *x*_*ij*_-comparing each data of the sequence, *p*-th *p* objects, *n*-the data length of the sequence, that is, the number of data.

The article "Optimization of Management Structure and Resource Coordination Management Method of Construction Enterprises under Urban Environmental Pollution" was published in 2022. Journal: J Environ Public Health.

*X*-data value, *i*-the *i*th object, *t*-period *t*, *j*-*j*th indicator; when *i* = 0, *x*_*ij*_-comparing each data of the sequence, *p*-th *p* objects, the *n*-the data length of the sequence, that is, the number of data.

Calculate the absolute dispersion value: record the absolute value of the difference between the value of each period of the *k*-th comparison sequence (*k* = 1, 2, ..., *P*) and the corresponding period of the reference value sequence as:

(5) $$\begin{array}{c} {⊳}_{OR}\left(t\right)=\left|x_{o}\left(t\right)-x_{R}\left(t\right)\right|. \end{array}$$

For the *k*-th comparison sequence, record the minimum and maximum numbers of *n*⊳__*OR*(*t*)__ as ⊳__*OR*__(min) and ⊳__*OR*__(max), respectively. For the *P* comparison columns, the smallest of the *P*⊳__*OR*__(min)'s is ⊳(min), and the largest of the *P*⊳__*OR*__(max)′s is ⊳(max). In this way, ⊳(min) and ⊳(max) are the smallest and largest of the absolute values of all *P* comparison sequences in each period, respectively. Obviously,

(6) $$\begin{array}{c} \Delta \left(\min\right)=\underset{j}{\min}\left[\underset{i}{\min\Delta_{OK}\left(t\right)}\right], \end{array}$$

(7) $$\begin{array}{c} \Delta \left(\max\right)=\underset{j}{\max}\left[\underset{i}{\max\Delta_{OK}\left(t\right)}\right]. \end{array}$$

Calculation of correlation coefficient: According to the theory and method of grey correlation analysis, the correlation degree between the *k*-th comparative sequence and the reference sequence in period *t* can be calculated by the formula:

(8) $$\begin{array}{c} \zeta_{OR}\left(t\right)=\frac{⊳\left(\min\right)+\rho ⊳\left(\max\right)}{{⊳}_{OK}\left(t\right)+\rho ⊳\left(\max\right)}. \end{array}$$

Calculate the degree of association, and then calculate the degree of association between the *i*th evaluated object and the optimal reference sequence according to formula:

(9) $$\begin{array}{c} r_{i}=\frac{1}{p}\sum_{j=1}\zeta_{ij}. \end{array}$$

The formula for calculating the comprehensive evaluation coefficient *Ei* is:

(10) E=iri×100.

In fact, *Ei* has the same meaning as relevance *r*_*i*_. The scale factor is set to 100, just to be consistent with people's accustomed grading method.

Since *r*_*i*_ reflects the degree of correlation between the *i*th evaluated object and the standard evaluation sequence x_0*i*_, if *Ei* >*Ej* , it means that the *i*th sample is better than the *j*th sample. Therefore, according to {*Ei*}, the objects to be evaluated can be sorted and comparatively analyzed.

1. Determine the reference sequence;
2. Perform dimensionless processing on the actual value of each indicator;
3. Find the two-level maximum difference Δ(max) and the two-level minimum difference Δ(min);
4. Calculate the correlation coefficient and correlation degree
5. Calculate the comprehensive evaluation coefficient *Ei*;
6. According to {*Ei*}, the objects to be evaluated can be sorted and comparatively analyzed.

The article "Optimization of Management Structure and Resource Coordination Management Method of Construction Enterprises under Urban Environmental Pollution" was published in 2022. Journal: J Environ Public Health.

### 3.2. Principal Component Analysis

First, an evaluation index system is established according to the content, and the variable matrix *X* of the index system is established, which is composed of *n* questionnaire samples and *p* index samples. The matrix form is as follows:

(11) $$\begin{array}{c} X=\left[\begin{array}{c} X_{1}^{T}\\ X_{2}^{T}\\ \vdots \\ X_{N}^{T} \end{array}\right]=\left[\begin{array}{cccc} x_{11} & x_{12} & \cdots & x_{1p}\\ x_{21} & x_{22} & \cdots & x_{2p}\\ \vdots & \cdots & \cdots & \vdots \\ x_{n1} & x_{n2} & \cdots & x_{np} \end{array}\right]. \end{array}$$

In order to eliminate the influence of the dimension and order of magnitude of the original data, the indicators are usually dimensionless, and the *Z*-score method is commonly used as follows:

(12) $$\begin{array}{c} Z=\frac{\left(x_{ij}-{\bar{x}}_{j}\right)}{\sqrt{\mathrm{var}\left(x_{j}\right)}},\;\left(i=1,2,\ldots ,n;\;j=1,2,\ldots ,p\right). \end{array}$$

Get the normalized data array:

(13) $$\begin{array}{c} Z_{ij}={\left(Z_{ij}\right)}_{n\times p}. \end{array}$$

The sample values are:

(14) $$\begin{array}{c} {\bar{x}}_{j}=\sum_{i=1}^{n}\frac{x_{ij}}{n}. \end{array}$$

The sample variance is:

(15) $$\begin{array}{c} \mathrm{var}\left(x_{ij}\right)=\frac{{\sum_{i=1}^{n}\left(x_{ij}-{\bar{x}}_{j}\right)}^{2}}{\left(n-1\right)}. \end{array}$$

Finding the correlation coefficient matrix of the standardized data, let *r*_*ij*_=1/*n* − 1∑*Z*_*ij*_ × *Zij*, namely,

(16) $$\begin{array}{c} r_{ij}=\frac{1}{n-1}x\sum_{i=1}^{n}\left[\left(x_{ij}-{\bar{x}}_{j}\right)/\sqrt{\mathrm{var}\left(x_{j}\right)}\right]\left[\left(x_{ik}-{\bar{x}}_{k}\right)/\sqrt{\mathrm{var}\left(x_{j}\right)}\right]. \end{array}$$

These have to be

(17) $$\begin{array}{c} R={\left(r_{ij}\right)}_{p\times p}. \end{array}$$

Since *r*_*jj*_=1; *r*_*ik*_=*r*_*ki*_ that is, *R* is a symmetric matrix, all elements on the diagonal are 1.

Since *r*_*jj*_=1; *r*_*ik*_=*r*_*ki*_ so *R* is a symmetric matrix, all elements on the diagonal are 1.

From the characteristic equation |*λI*_*P*_ − *R*|=0, *p* characteristic roots can be obtained:

(18) $$\begin{array}{c} \lambda_{g}=\left\{\lambda_{1},\lambda_{2},\cdots ,\lambda_{p}\right\}\left(\text{g}=1\text{,}2\text{,}\ldots ,\text{p}\right). \end{array}$$

And arrange them in order of size: *λ*_1_ ≥ *λ*_2_ ≥ ⋯≥*λ*_*p*_ ≥ 0, where each feature root corresponds to a feature vector *U*_*g*_(*U*_*g*_={*u*_*g*1_, *u*_*g*2_, *u*_*gp*_}). The SPSS software will directly export the eigenvalues and determine the principal components according to the eigenvalues. At the same time, the selected principal components are compared and determined according to the gravel diagram in the SPSS software to ensure the reliability of the selected principal components. According to the method of principal component extraction, remember to select the principal component as: *Y*_1_, *Y*_2_, ⋯, *Y*_*m*_, then:

(19) $$\begin{array}{c} \left\{\begin{array}{c} Y_{1}=u_{11}x_{1}+u_{12}x_{2}+\cdots +u_{1p}x_{p},\\ Y_{2}=u_{21}x_{1}+u_{22}x_{2}+\cdots +u_{2p}x_{p},\\ \vdots \\ Y_{M}=u_{m1}x_{1}+u_{m2}x_{2}+\cdots +u_{mp}x_{p}. \end{array}\right) \end{array}$$

Among them, *Y*_1_, *Y*_2_, ⋯, *Y*_*m*_ is the first principal component, the second principal component, the third principal component...the *m-*th principal component. The purpose of the principal component analysis is to find the linear combination of *X*_1_, *X*_2_, ⋯, *X*_*P*_, which is used to represent each principal component, obtain the score of the principal component through relevant mathematical calculations, and then weight to obtain the comprehensive score of all principal components as the basis for evaluation. Calculate the score *F*_*i*_ of *n* samples on *m* principal components:

(20) $$\begin{array}{c} F_{i}=u_{1i}X_{1}+u_{2i}X_{2}+\cdots +u_{pi}X_{p}\left(\text{i}=1,2,\ldots ,\text{m}\right). \end{array}$$

The weight of each index can be obtained by weighting the comprehensive index score *F*.

(21) $$\begin{array}{c} F=\sum_{i=1}^{m}w_{i}F_{i}, \end{array}$$

(22) $$\begin{array}{c} w_{i}=a_{i}=\frac{\lambda_{i}}{\sum_{m=1}^{p}\lambda_{m}}. \end{array}$$

The evaluation score can be comprehensively determined by combining the index weight and the score of each index.

The article "Optimization of Management Structure and Resource Coordination Management Method of Construction Enterprises under Urban Environmental Pollution" was published in 2022. Journal: J Environ Public Health.

## 4. Analysis of Optimization of Management Structure of Construction Enterprises and Coordinated Management of Resources under Urban Environmental Pollution

### 4.1. The Status of Green Buildings in Construction Enterprises

From 2010 to 2017, the number of green building evaluation and labeling projects in China increased year by year, and only the number of green building evaluation and labeling projects in 2018 was relatively lower than the previous year. As can be seen from Figure 4, the growth rate reached 193.90% in 2011. Although the growth rate decreased from 2011–2015, the number of green building evaluation and identification projects has been increasing, indicating that the country is increasingly concerned about urban green buildings. Therefore, construction companies need to optimize their own business structure and coordinate the management of resources, so that construction companies can follow national policies and develop in the long run, as shown in Figure 4.

The researchers mainly selected more construction majors, followed by energy majors, and fewer other majors. From the perspective of age, the 25–29 age group is the largest, followed by the 30–34 age group, then the 20–24 age group, and finally the 35-year-old and above; the average age of the surveyed green building-related personnel is relatively young, this is because the evaluation work related to green building in China has only developed in recent years. From the perspective of the respondents' cognition and understanding of green building evaluation systems at home and abroad, all the surveyed people have some understanding of ESGB. Among other green building evaluation systems, LEED in the United States has the largest number of people, followed by BREEAM, ESGB, CASBEE, CEHRS, DGNB, GOBAS, HK-BEAM, SBTOOL, EEWH. It can be seen that few people understand some green building evaluation systems in China, as shown in Figure 5.

### 4.2. Indicator Construction

In order to analyze the management structure optimization and resource coordination management method of construction enterprises under the urban environmental pollution, the index system should be established first, and then the in-depth analysis and research should be carried out. By establishing two-level indicators, the first-level indicators include enterprise mechanism (A), talent quality (B), management performance (C), operation management (D), and resource coordination management (E); the second-level indicators include management system (A1), talent atmosphere (A2), corporate culture (A3), employee quality (B1), employee capability (B2), employee qualification compliance rate (C1), key talent loss rate (C2), product quality qualification rate (C3)), energy conservation management (D1), greening management (D2), waste management (D3), intelligent system management (D4), building main energy conservation (E1), energy system planning and utilization (E2), renewable energy utilization (E3), and the impact of energy consumption on the environment (E4), as shown in Table 1.

### 4.3. Index Analysis of Management Structure Optimization and Resource Coordination Management Methods of Construction Enterprises

Among the first-level indicators, resource coordination management (E) has the largest weight, with a weight of 0.24, followed by operation management (D), enterprise mechanism (A), talent quality (B), and management performance (C), with a weight of 0.22, 0.2, 0.19, 0.15. As shown in Figure 6, the secondary indicators have the largest weight value of energy system planning and utilization (E2), with a weight of 0.0727, followed by renewable energy utilization (E3), enterprise employee qualification rate (C1), waste management (D3), greening management (D2), energy saving management (D1), main building energy saving (E1), impact of energy consumption on the environment (E4), management system (A1), corporate culture (A3), employee ability (B2), qualified product quality rate (C3), intelligent system management (D4), key talent loss rate (C2), talent atmosphere (A2), and staff quality (B1), as shown in Table 2.

The article "Optimization of Management Structure and Resource Coordination Management Method of Construction Enterprises under Urban Environmental Pollution" was published in 2022. Journal: J Environ Public Health.

The weight values of the secondary indicators are not much different, and the weight value is about 0.6. Energy system planning and utilization (E2) is the most important, with a weight value of 0.0727, and the least important is employee quality (B1), with a weight value of 0.051, and the difference between the two weight values is 0.0217. Under urban environmental pollution, the optimization of the management structure of construction enterprises and the coordinated management of resources are relatively important, as shown in Figure 6.

In the index, the combined value of CMIN/DF is 4, and the boundary value is less than 5, which judges the fruit to conform to the line; If the fitting value of GFI is 1.1, the fitting value of AGFI is 0.98, and the fitting value of RFI is 0.98 is 0.99, all meet the critical value greater than 0.9, so the judgment result is consistent; the PNFI external fitting value is 0.93, and the critical value is greater than 0.5, so the judgment result is consistent; the RMSEA fitting value is 0.02, and the critical value is less than 0.08, So the judgment result is in line. It shows that the model fitting effect is good, and the model is established, as shown in Table 3.

From Table 4, we can see that the estimated value of the standardized coefficients between the management structure of construction enterprises and the five structural variables is the degree of the direct impact of each index on the management structure of construction enterprises. At the 5% significant level, the *p*-values between the enterprise mechanism (A), management performance (C), talent quality (B), operation management (D), resource coordination management (E) and the construction enterprise management structure path are all less than 0.05, these five first-level indicators will affect the operation of construction enterprises. The standardized estimated value of resource coordination management (E) is the largest, which is 0.47, indicating that resource coordination management (E) has the greatest impact on the operation of construction enterprises; followed by operation management (D), enterprise mechanism (A), talent quality (B), management performance (C), the standardized estimates are 0.46, 0.45, 0.42, and 0.4, respectively, indicating that the most important thing for the operation of the cultural industry is the improvement of resource coordination management (E), as shown in Table 4.

The article "Optimization of Management Structure and Resource Coordination Management Method of Construction Enterprises under Urban Environmental Pollution" was published in 2022. Journal: J Environ Public Health.

In enterprise mechanism (A), the influence coefficients of the management system (A1), talent atmosphere (A2), and corporate culture (A3) are 0.812, 0.756, and 0.894, respectively, indicating that corporate culture (A3) and management system (A1) are relatively important reasons that affect industrial resources. In talent quality (B), the coefficients of employee quality (B1) and employee ability (B2) are 0.762 and 0.867, respectively, indicating that employee ability (B2) has the greatest impact on it, and the enterprise attention should be paid to the introduction of talents to improve the comprehensive ability of employees. In the management performance (C), the influence coefficients of the employee qualification rate (C1), the key talent loss rate (C2), and the product quality qualification rate (C3) are respectively, 0.866, 0.756, 0.857, indicating that the employee qualification rate (C1) is more important to management performance (C), so construction companies should train employees to improve the employee qualification rate, and at the same time control product quality. In (D), the influence coefficients of energy saving management (D1), greening management (D2), waste management (D3), and intelligent system management (D4) are 0.932, 0.927, 0.911, and 0.901, respectively. The impact of green building is relatively large, indicating that construction companies should improve and optimize green buildings, closely follow national policies, and develop in the long run. In resource coordination management (E), building main body energy conservation (E1), energy system planning and utilization (E2), the utilization of renewable energy (E3), and the impact of energy consumption on the environment (E4) are 0.897, 0.894, 0.899, and 0.898, respectively, indicating that the utilization of renewable energy (E3) has the greatest impact on it, and the main building energy conservation (E1)), energy system planning and utilization (E2), and the impact of energy consumption on the environment (E4) also have a relatively large impact on resource coordination management (E). Recyclability is still a concept of a continuous process, as shown in Table 5.

The article "Optimization of Management Structure and Resource Coordination Management Method of Construction Enterprises under Urban Environmental Pollution" was published in 2022. Journal: J Environ Public Health.

It can be seen from Table 5 that in terms of enterprise mechanism (A), corporate culture (A3), and management system (A1) are relatively important factors affecting industrial resources; in terms of talent quality (B), employee ability (B2) has the greatest impact on it and enterprises should pay attention to the introduction of talents and improve the comprehensive ability of employees; in terms of management performance (C), construction enterprises should train employees, improve the qualification rate of employees, and also control product quality; in operation management (*D*)), construction enterprises should improve and optimize green buildings, follow national policies, and develop in the long run; in terms of resource coordination management (E), construction enterprises should continue to deepen the concept of green buildings, and also strengthen the recycling of green building materials and equipment. Recycling is still a continuous concept.

From Figure 7, we can see whether the degree of direct influence of the estimated value of the standardized coefficient between the first-level index and the second-level index is significant. At the 5% significant level, the *P* values between the paths of the secondary indicators and the primary indicators are all less than 0.05, indicating that the path of structural variables and each indicator variable has a significant impact.

## 5. Conclusions

Construction enterprises should establish sound organizational structures and green construction management systems and systems. To improve employees' awareness of green building management and strengthen the management of professional responsibilities of managers, the purpose of managing green building organizations is to establish a green building management system. Managers should have a clear division of labor, standardize the positions of greenfield managers and supervisors, and effectively guarantee and promote the implementation of green projects. Provide regular training and material incentives to encourage employees to deepen their understanding of green building or select outstanding employees to learn green building professional knowledge to improve their overall quality. Vigorously develop technologies related to green construction technology in construction technical standards, and formulate corresponding implementation measures. The classification and recycling of construction waste is an optimized plan for material saving measures, and the green construction of construction projects should focus on five aspects: environmental protection, water resource protection and water resource utilization, material resource protection and utilization, energy saving and energy utilization, and land protection and land resource protection and each aspect should be evaluated. In order to prevent ineffective project supervision, corresponding measures have been formulated to strengthen the supervision of each link.

The article "Optimization of Management Structure and Resource Coordination Management Method of Construction Enterprises under Urban Environmental Pollution" was published in 2022. Journal: J Environ Public Health.

The experimental data used to support the findings of this study are available from the corresponding author upon request.

## Figures and Tables

**Figure 1:** Current status of environmental protection management.

**Figure 2:** Characteristics of urban environmental pollution caused by construction products.

**Figure 3:** Optimization of construction enterprise management structure under urban environmental pollution.

**Figure 4:** Number of green building evaluation and labeling projects.

**Figure 5:** Survey people's understanding of green building evaluation systems at home and abroad.

**Figure 6:** Secondary indicator weights.

**Figure 7:** Comparison of *P* values and critical values.

**Table 1:** Indicator system.

First-level indicator	Secondary indicators
Enterprise mechanism (A)	Management system (A1)
	Talent atmosphere (A2)
	Corporate culture (A3)

Talent quality (B)	Staff quality (B1)
	Employee competency (B2)

Management performance (C)	Employee qualification compliance rate (C1)
	Key brain attrition rate (C2)
	Product quality pass rate (C3)

Operation management (D)	Energy conservation management (D1)
	Greening management (D2)
	Waste management (D3)
	Intelligent system management (D4)

Resource coordination management (E)	Building main body energy saving (E1)
	Energy system planning and utilization (E2)
	Renewable energy utilization (E3)
	Environmental impact of energy consumption (E4)

**Table 2:** Indicator weights.

First-level indicator	Weight	Secondary indicators	Weight
Enterprise mechanism (A)	0.2	Management system (A1)	0.063
		Talent atmosphere (A2)	0.056
		Corporate culture (A3)	0.063

Talent quality (B)	0.19	Staff quality (B1)	0.051
		Employee competency (B2)	0.063

Management performance (C)	0.15	Employee qualification compliance rate (C1)	0.066
		Key brain attrition rate (C2)	0.057
		Product quality pass rate (C3)	0.0593

Operation management (D)	0.22	Energy conservation management (D1)	0.064
		Greening management (D2)	0.065
		Waste management (D3)	0.066
		Intelligent system management (D4)	0.059

Resource coordination management (E)	0.24	Building main body energy saving (E1)	0.0635
		Energy system planning and utilization (E2)	0.0727
		Renewable energy utilization (E3)	0.068
		Environmental impact of energy consumption (E4)	0.0635

The article "Optimization of Management Structure and Resource Coordination Management Method of Construction Enterprises under Urban Environmental Pollution" was published in 2022. Journal: J Environ Public Health.

**Table 3:** Overall model fitting results.

Adaptation indicator	CMIN/DF	GFI	AGFI	RFI	PNFI	RMSEA
Critical value	<5	>0.9	>0.9	>0.9	>0.5	<0.08
Fitted value	4	1.1	0.98	0.99	0.93	0.02
Judgement result	Meets	Meets	Meets	Meets	Meets	Meets

**Table 4:** Summary of the calculation results of the impact parameters of the first-level indicators on the management structure of construction enterprises.

Project path			Standardized estimates	Standard deviation	Critical ratio	*P* value
Business structure	<--	Enterprise mechanism (A)	0.45	0.09	2.25	0.032
Business structure	<--	Talent quality (B)	0.42	0.07	2.21	0.029
Business structure	<--	Management performance (C)	0.4	0.067	2.32	0.034
Business structure	<--	Operation management (D)	0.46	0.092	2.43	0.03
Business structure	<--	Resource coordination management (E)	0.47	0.094	1.53	0.022

**Table 5:** Summary of the calculation results of the influence parameters of the secondary indicators on the primary indicators.

Project path			Standardized estimates	Standard deviation	Critical ratio	*P* value
A	<--	A1	0.812	0.03	16.85	0.024
A	<--	A2	0.756	0.05	25.64	0.029
A	<--	A3	0.894	0.034	27.65	0.034
B	<--	B1	0.762	0.029	24.59	0.023
B	<--	B2	0.867	0.016	24.19	0.0136
C	<--	C1	0.866	0.018	19.86	0.0101
C	<--	C2	0.756	0.027	16.73	0.0131
C	<--	C3	0.857	0.057	30.18	0.002
D	<--	D1	0.932	0.017	29.67	0.014
D	<--	D2	0.927	0.18	22.29	0.025
D	<--	D3	0.911	0.019	26.35	0.0291
D	<--	D4	0.901	0.033	29.68	0.0171
E	<--	E1	0.897	0.055	16.28	0.021
E	<--	E2	0.894	0.058	18.44	0.0104
E	<--	E3	0.899	0.034	19.25	0.0341
E	<--	E4	0.898	0.029	20.23	0.024

## Data Availability

The experimental data used to support the findings of this study are available from the corresponding author upon request.
